The article "Dysregulation of Survivin-Targeting microRNAs in Autoimmune Diseases: New Perspectives for Novel Therapies" was retracted in 2023. Reason: concerns about the authorship.

# Dysregulation of Survivin-Targeting microRNAs in Autoimmune Diseases: New Perspectives for Novel Therapies

**DOI:** 10.3389/fimmu.2022.839945

**Published:** 2022-03-03

**Authors:** Navid Shomali, Marwah Suliman Maashi, Behzad Baradaran, Amin Daei Sorkhabi, Aila Sarkesh, Hamed Mohammadi, Maryam Hemmatzadeh, Faroogh Marofi, Siamak Sandoghchian Shotorbani, Mostafa Jarahian

**Affiliations:** ^1^ Immunology Research Center, Tabriz University of Medical Sciences, Tabriz, Iran; ^2^ Department of Immunology, Faculty of Medicine, Tabriz University of Medical Sciences, Tabriz, Iran; ^3^ Student Research Committee, Tabriz University of Medical Sciences, Tabriz, Iran; ^4^ Medical Laboratory Technology Department, Faculty of Applied Medical Sciences, King Abdulaziz University, Jeddah, Saudi Arabia; ^5^ Non-Communicable Diseases Research Center, Alborz University of Medical Sciences, Karaj, Iran; ^6^ Department of Immunology, School of Medicine, Alborz University of Medical Sciences, Karaj, Iran; ^7^ German Cancer Research Center, Toxicology and Chemotherapy Unit (G401), Heidelberg, Germany

**Keywords:** survivin, microRNA, autoimmune disease, rheumatoid arthritis (RA), inflammatory bowel disease (IBD), psoriasis, systemic lupus erythematosus (SLE), and multiple sclerosis (MS)

## Abstract

It has been well established that the etiopathogenesis of diverse autoimmune diseases is rooted in the autoreactive immune cells’ excessively proliferative state and impaired apoptotic machinery. Survivin is an anti-apoptotic and mitotic factor that has sparked a considerable research interest in this field. Survivin overexpression has been shown to contribute significantly to the development of autoimmune diseases *via* autoreactive immune cell overproliferation and apoptotic dysregulation. Several microRNAs (miRNAs/miRs) have been discovered to be involved in survivin regulation, rendering the survivin-miRNA axis a perspective target for autoimmune disease therapy. In this review, we discuss the role of survivin as an immune regulator and a highly implicated protein in the pathogenesis of autoimmune diseases, the significance of survivin-targeting miRNAs in autoimmunity, and the feasibility of targeting the survivin-miRNA axis as a promising therapeutic option for autoimmune diseases.

## Introduction

The complex etiopathogenesis of various autoimmune conditions has prompted researchers to investigate the molecular basis and factors associated with the high proliferative and apoptosis-resistant state of implicated cells (1, 2). In this way, research into anti-apoptotic factors and their potential role in developing various pathological conditions, including malignancies and autoimmune diseases, has offered a promise for future clinical approaches. Survivin, a member of the inhibitor of apoptosis protein (IAP) family, has been found to enhance cell survival *via* regulating mitotic and anti-apoptotic pathways (3, 4). Besides, survivin is endowed with regulative roles in immune cells development and their competent function (5, 6). However, these impacts appear unwanted in autoimmune conditions, indicating that an aberrant survivin expression profile is a fundamental etiologic factor and therapeutic target. Upregulated survivin expression in autoreactive immune cells from patients with various autoimmune diseases has been evidenced in this context. Further investigation into the regulatory pathways of survivin mRNA in these cells has shown the emerging role of survivin-targeting miRNAs in the maintenance of autoreactivity (7, 8).

The article "Dysregulation of Survivin-Targeting microRNAs in Autoimmune Diseases: New Perspectives for Novel Therapies" was retracted in 2023. Reason: concerns about the authorship.

MicroRNAs (miRNAs/miRs) are endogenous non-coding RNAs that bind to perfect or imperfect complementary sequences in 3′-untranslated regions (3′-UTRs) of protein-coding mRNAs to regulate degradation or translational repression (9–11). Multiple survivin-targeting miRNAs have been discovered, with the potential to either directly bind the 3′-UTR of survivin mRNA or to indirectly influence the pathways that alter survivin expression as a downstream target (12). Although research into the relevance of these miRNAs in autoimmune conditions is still in its infancy, their validated implication in cancer studies opens up a new avenue for evaluating miRNA-based therapeutic approaches to regulate survivin expression.

This review will discuss the structure and function of survivin under healthy settings and its implications in the pathogenesis of autoimmune diseases. Also, we will go into detail on the regulatory roles of individual miRNAs in certain autoimmune diseases and the clinical perspectives of targeting the survivin-miRNA axis.

## Structure and Function of Survivin

Survivin is the smallest member of the IAP family found for the first time in 1997 while hybridization screening of a human genomic library (13). The baculoviral IAP repeat-containing 5 (BIRC5) gene, which encodes survivin, is mapped to the telomeric region of chromosome 17q25 and is reversely complementary to the effector cell protease receptor-1 (EPR-1) gene (14). BIRC5 encodes wild type (WT) survivin as well as five alternative splice variants: survivin-ΔEx3 (with deletion of exon 3), survivin-2B (with additional exon), survivin-3B (with five exons), survivin 2α (with two exons), and survivin 3α (with two exons) (15). Among these isoforms, survivin-WT, survivin-2B, and survivin-ΔEx3 account for about 98% of survivin mRNAs. Survivin is a 16.5 kDa protein with 142 amino acid residues consisting of an N-terminal Zn^2+^-binding BIR domain and a 65 Å amphipathic C-terminal alpha-helical alpha coiled‐coil domain that replaces the IAP-specific RING finger domain, with amino acid residues 15-89 and 100-140, respectively. Survivin forms a homodimer by a symmetrical interaction between two survivin monomers across the dimerization interface, which consists of amino acid residues 6-10 and 89-102. This dimeric structure is essential for survivin protein stabilization and functionality by establishing non-polar interactions between residues (16, 17). Mechanistically, the single zinc finger folds BIR domain is implicated in the anti-apoptotic activities of survivin. Conversely, the alpha-helix domain is involved in nuclear exportation and protein-protein interaction, specifically interaction with microtubular structures, which are essential for cell division (18). Additionally, dimer interfaces enable survivin to establish a stable homodimeric state that appears to be involved in mitotic activity, whilst survivin’s monomeric state is primarily attributed to its anti-apoptotic properties (19, 20).

The article "Dysregulation of Survivin-Targeting microRNAs in Autoimmune Diseases: New Perspectives for Novel Therapies" was retracted in 2023. Reason: concerns about the authorship.

The multiple functions of survivin are impacted by reversible dimerization, posttranslational modifications, and subcellular localization (21). The subcellular localization of survivin isoforms varies, with some being extracellular and others being intracellular. Extracellular survivin has been demonstrated to be released by cancer cells, and exosomally delivered to cancer cells, promoting tumorigenesis (22). On the other hand, intracellular isoforms are cytoplasmic survivin or mitochondrial survivin, which inhibit apoptosis and have a cytoprotective role in cancer cells. Others are nuclear survivin, which regulates cell division (23). Taken together, survivin is mainly endowed with the dual role of mitotic and anti-apoptotic regulation.

As a negative apoptosis regulator, Survivin is involved in several anti-apoptotic pathways, which may be characterized as caspase-dependent and caspase-independent apoptosis inhibition. In this way, survivin directly inhibits the terminal effector enzymes caspase-3, caspase-7, and caspase-9, enabling cells to resist apoptosis triggered by particular stimuli (24, 25). Caspase-9 has also been inhibited indirectly by binding the survivin-hepatitis B X-interaction protein (HBXIP) complex to procaspase-9, therefore blocking apoptosis triggered by the mitochondria/cytochrome *c* pathway (26). Furthermore, survivin interacts with cofactor molecules, namely X-linked IAP (XIAP). The formation of the survivin-XIAP complex shelters XIAP from proteasomal degradation and contributes to the inhibition of caspase-9-dependent apoptosis (27). On the other hand, survivin interacts with intermediate apoptotic proteins, such as the second mitochondria-derived activator of caspase (SMAC/DIABLO), and this interaction indirectly restricts caspase activation. Survivin colocalizes with SMAC, disrupting the physical association of SMAC and inhibiting cytochrome *c*-dependent apoptosis (28) (**Figure 1**). Ultimately, survivin inhibits various caspase-independent pathways through pro-apoptotic proteins such as apoptosis-inducing factor (AIF). Survivin binds to AIF in the mitochondria and hinders its nuclear translocation, wherever it triggers DNA fragmentation and so apoptosis (29).

The article "Dysregulation of Survivin-Targeting microRNAs in Autoimmune Diseases: New Perspectives for Novel Therapies" was retracted in 2023. Reason: concerns about the authorship.

**Figure 1:** Survivin: Key Regulator of Mitosis and Apoptosis. The death receptor (extrinsic) or mitochondrial (intrinsic) pathways can both trigger apoptosis. Both the extrinsic and intrinsic mechanisms function through caspase-8 and caspase-9. Survivin co-immunoprecipitates with caspases-3, -8, and -9 and reduces apoptosis triggered by these caspases, showing that survivin is also a caspase inhibitor. Survivin inhibits Smac/DIABLO activity and may aid the action of other IAPs such as XIAP and HBXIP. XIAP is a potent apoptosis inhibitor that binds directly with caspases and suppresses them. In the nucleus, survivin interacts with aurora B kinase and the inner centromere protein (INCEP) to regulate chromosomal alignment during mitosis as part of the chromosomal passenger complex (CPC). Survivin can also enhance cell motility by activating Akt and increasing the expression of integrin alpha-5. AKT, serine/threonine kinase; AURKB, Aurora B kinase; Bax, bcl-2-like protein 4; CPC, The chromosomal passenger complex; Cyst, cytochrome c; FADD, Fas-associated protein with death domain; HBIXP, Hepatitis B X-interacting protein; SMAC, Second mitochondria-derived activator of caspases; TRADD, Tumor necrosis factor receptor type 1-associated death domain; XIAP, X-linked inhibitor of apoptosis protein.

Survivin synthesis, expression, and degradation are cell cycle-dependent in normal tissues; they are abundantly expressed during the G2/M phase and dramatically drop during the G1 phase (30). Survivin also operates in a restricted time frame during metaphase and anaphase, indicating a significant mitotic regulation role for survivin. In this respect, survivin is an integral part of the chromosomal passenger complex (CPC) that directs the CPC to kinetochores during metaphase to lead proper chromosome orientation preceding anaphase. Its enzymatic subunit Aurora-B kinase interacts with the spindle checkpoint tension sensor BubR1 to detect and dissociate misaligned chromosomes (31). Then, during anaphase, this complex translocates to midzone microtubules and regulates central spindle assembly and cytokinesis (32). Furthermore, it has been demonstrated that an additional survivin subcellular pool is intimately associated with polymerized tubulin and is implicated in microtubule synthesis and dynamics during mitosis (33).

The article "Dysregulation of Survivin-Targeting microRNAs in Autoimmune Diseases: New Perspectives for Novel Therapies" was retracted in 2023. Reason: concerns about the authorship.

## Participation of Survivin in the Immune System

Survivin is involved in various developmental and functional features of adaptive and innate immune cells, owing to its mitotic and anti-apoptotic roles. Several studies have outlined survivin expression in tissues with proliferative cells, such as the thymus, and its significance in thymocyte maturation and development of T-lymphocytes (34). In this respect, selective survivin deletion has been established to impair the transition of double negative to double-positive thymocytes, leading to a decrease in mature CD4^+^ and CD8^+^ T cell subsets (5). Survivin deletion significantly impacts T cells’ homeostatic and mitogen-induced proliferation than apoptotic T cell death. It impairs the development of a functional T cell receptor, leading to a disrupted considerably immune response upon antigen exposure (35). Unlike other terminally differentiated cells, survivin is upregulated in activated T cells following OX40 activation of PKB (Akt), enabling for persistent T cell expansion and phenotypic transitions like the development of effector and memory CD4^+^ T cells, the maintenance of virus-specific CD8^+^ memory T cells, and differentiation into regulatory CD25^+^FOXP3^+^CD4^+^ and follicular CXCR5^+^BCL6^+^ T cells (36–38). Survivin also boosts T helper 2 (Th2) immune response and compensates for OX40 co-stimulatory deficit, underlies asthmatic allergic reactions (39). Moreover, survivin has been shown to regulate metabolic adaptation in interferon-gamma (IFN-γ) producing CD4^+^ T cells requisite for effector function. It directly interacts with interferon regulatory factor-1 (IRF1) and recruits to chromatin regulatory regions to restrict the expression of the glycolytic enzyme 6-phosphofructo-2-kinase/fructose-2,6-bisphosphatase 3 (PFKFB3) and encourage glucose metabolism *via* the pentose phosphate pathway (40).

The sustained expression of survivin has been exhibited throughout the small pre-B cell stage in the mice model, proceeded by downregulation in immature B cells of the bone marrow so that it is no longer detectable in either naive B cells in secondary lymphoid organs or recirculating B cells in the bone marrow. Survivin upregulation in proliferative germinal center (GC) B cells impairs antibody class switching and plasma cell development. Accordingly, the survivin-deficient mice model was shown to have defective plasma cells and immunoglobulin (Ig) G1 positive cell formation, rendering that incapable of mounting a humoral immune response (6). However, survivin overexpression in autoimmune disease contributes to escape apoptosis in autoreactive B cells, preserving autoreactive lymphocytes that would otherwise be eliminated by apoptosis (41). These findings indicate that survivin has the potential to be a therapeutic target in autoimmune diseases (42).

The article "Dysregulation of Survivin-Targeting microRNAs in Autoimmune Diseases: New Perspectives for Novel Therapies" was retracted in 2023. Reason: concerns about the authorship.

Survivin plays a pivotal role in antigen presentation through regulating the maturation of dendritic cells (DCs) and the formation of antigen-presenting machinery components such as major histocompatibility complex (MHC) class II (43). In this regard, survivin inhibits the DC-committed progenitor cells’ apoptosis, optimizing their survival, while also up-regulating co-stimulatory molecules CD80/CD86 and MHC class II (44). Besides, survivin overexpression has been demonstrated to increase proliferation and mediate non-classical antigen presentation on monocyte-derived DCs through the CD1a receptor (45). Moreover, survivin is expressed by other innate immune cells, including immature neutrophils. It is essential for their maturation and expansion during granulocytopoiesis and their persistent inflammatory response, mediated by survivin re-expression-induced apoptosis inhibition (46, 47). Additionally, macrophages’ survivin expression in atherosclerotic events has dual regulatory anti-atherogenic effects. Survivin enhances macrophage recruitment in the arterial wall and plaque formation. Still, it is negatively regulated in the presence of oxidized lipid byproducts, which contribute to apoptotic cell death and plaque weakness (48, 49).

## Irregular Expression of Survivin-Specific microRNAs in Specific Autoimmune Disease

Survivin overexpression in various immunopathological conditions such as autoimmune diseases has opened up a new avenue to investigate its role as an etiologic and prognostic factor, diagnostic marker, and therapeutic target. Multiple studies have found aberrant survivin expression in rheumatoid arthritis (RA) (50), inflammatory bowel disease (IBD) (51), psoriasis (52), systemic Lupus erythematosus (SLE) (53), and multiple sclerosis (MS) (54). Survivin overexpression has been shown to significantly contribute to the etiopathogenesis of these conditions thanks to its mitotic and antiapoptotic properties. Also, multiple survivin-specific miRNAs with aberrant expression profiles have been identified in autoimmune diseases that play a central role in survivin regulation (**Table 1**). The specific consequences of these miRNAs in various autoimmune disorders will be discussed in the following parts.

The article "Dysregulation of Survivin-Targeting microRNAs in Autoimmune Diseases: New Perspectives for Novel Therapies" was retracted in 2023. Reason: concerns about the authorship.

**Table 1:** Dysregulation of Survivin-targeting microRNAs in various autoimmune diseases.

*Autoimmune disease*	*Profiled miRNAs*	*MiRNA expression status*	*Survivin regulation*	*reference*
*Rheumatoid arthritis*	miR-16	Upregulated in serum, PBMCs, peripheral blood, and synovial fluid	Survivin downregulation as a result of p53/survivin signaling pathway modulation and direct interaction between 3′-UTR of survivin mRNA and miRNA	(10, 55)
	miR-150	Downregulated in serum, upregulated in IL-17 releasing T cells	Survivin upregulation in colon adenocarcinoma cell line as a result of downregulated TP53, survivin downregulation in Burkitt’s lymphoma cell line	(56, 57)
	miR-34	Downregulated in synovial fibroblasts	Survivin upregulation as a result of downregulated E2F3	(58, 59)
	miR-203	Upregulated in synovial fibroblasts	Survivin downregulation as a result of targeting nuclear factor-kappa B (NF-κB) pathway, PI3K-Akt axis and E2F3	(60–62).
*Inflammatory bowel disease (IBD)*	miR-16	Upregulated in serum	Survivin upregulation as a result of targeting NF-κB pathway	(63, 64)
	miR-21	Upregulated in colon tissue and CD4^+^ T cells	Survivin upregulation as a result of downregulated PTEN expression	(65, 66).
*Psoriasis*	miR-20a-3p	Downregulated in psoriatic lesions and keratinocytes of psoriasis patients.	Survivin upregulation as a result of post-transcriptional suppression of SFMBT1	(67)
	miR-125b	Downregulated in keratinocytes	Survivin upregulation as a result of a positive feedback loop involving STAT3/SH3PXD2A-AS1/miR-125b/STAT3	(68)
*Systemic lupus erythematosus (SLE)*	miR-16	Downregulated in serum	Survivin upregulation	(69, 70)
	miR-203	Downregulated in serum	Survivin upregulation	(69, 70)
	miR-20a	Downregulated in serum	Survivin upregulation as a result of NF-κB pathway activation	(69, 71)
	miR-21	Upregulated in CD4^+^ cells	Survivin upregulation as a result of downregulated PTEN expression	(66, 72).
*Multiple sclerosis (MS)*	miR-708	Downregulated in CD4+ cells	Survivin upregulation as a result of direct interaction between 3′-UTR of survivin mRNA and miRNA	(73–75)
	miR-485	Downregulated in CD4^+^ cells	Survivin upregulation as a result of direct interaction between miRNA and 3′-UTR of survivin mRNA	(74, 75)
	miR-34a	Downregulated in CD4^+^ cells	Survivin upregulation as a result of direct interaction between 3′-UTR of survivin mRNA and miRNA	(73)

### Rheumatoid *Arthritis*

RA is a complicated, inflammatory condition marked by irreversible and progressive synovial hyperplasia leading to articular joint destruction. Although the precise etiology has remained unknown, the cross-talk between innate and adaptive immunity, environmental variables, genetics, and epigenetic modifications have been demonstrated to be implicated in the initiation and progression of RA (76). The implication of survivin in RA pathogenesis has been established. It is substantiated by the upregulation of survivin in serum (77), synovial fluid (50), and peripheral blood mononuclear cells (PBMCs) (7) of RA patients, underpinning its potential relevance as a diagnostic biomarker and prognostic indicator in these patients (78, 79). It is evidenced further by research that found elevated survivin expression in patients with juvenile idiopathic arthritis to contribute to polyarticular involvement and systemic disease progression (80). Survivin dysregulation in RA patients’ fibroblast-like synoviocytes directly contributes to impaired apoptosis regulation and augmented mitosis, which leads to aberrant proliferation, pannus formation, and the acquisition of an invasive phenotype (81). On the other hand, survivin promotes inflammatory responses in RA by multiple mechanisms, including: i. contributing to the development of highly relevant T cell subsets in RA pathogenesis such as T follicular helper (Tfh), Th1, and Th17 (38, 82), ii. increasing leukocyte recruitment by upregulation of adhesion molecules like α-chains of β2-integrins on their surface (83), iii. enhancing immune cells’ resistance to apoptosis and therefore perpetuating autoreactive lymphocytes (84), iv. contributing to the formation of RA-specific autoantibodies, rheumatoid factor, and anti-citrullinated peptide antibodies (85).

The article "Dysregulation of Survivin-Targeting microRNAs in Autoimmune Diseases: New Perspectives for Novel Therapies" was retracted in 2023. Reason: concerns about the authorship.

Recent studies have convincingly emphasized the significance of dysregulation of the miRNA expression pattern in the pathophysiology of RA (86). Several miRNAs have been identified to bind to a specific sequence of survivin-coding mRNA or multiple binding sites at 3′‐UTR of survivin mRNA (12). To elaborate, miR-16 is overexpressed in RA patients’ serum, PBMCs, peripheral blood, and synovial fluid (87, 88). It has been established to either directly target survivin or modulate the p53/survivin signaling pathway. In this regard, a regulatory loop exists between miR-16 and p53 in which miR-16 downregulates p53 while p53 simultaneously up-regulates miR-16 and downregulates survivin, demonstrating that miR-16 indirectly regulates survivin expression by interacting with p53 (55). MiR-150 is another miRNA that is downregulated in serum but elevated in interleukin (IL)-17 releasing T cells of RA patients (56, 57). The specific influence of miR-150 on survivin expression has not been thoroughly elucidated. There are intriguing discoveries that it can downregulate the TP53 gene encoding p53, leading to survivin upregulation in colon adenocarcinoma cell lines. In contrast, it was demonstrated to downregulate survivin expression in Burkitt’s lymphoma cell line (89, 90). Furthermore, miR-34a is another survivin-specific miRNA that has been shown to be downregulated in synovial fibroblasts of RA patients (59). Survivin is downregulated by miR-34a relying upon multiple pathways. First, miR-34a directly targets and downregulates E2F3, leading to survivin downregulation as E2F3 is responsible for binding to the survivin promoter and enhancing survivin transcription (58). Second, miR-34a promotes the repression of transcriptional factor MYCN expression, which binds to and regulates the survivin promoter (91). Third, miR-34a alters survivin expression *via* interacting with the phosphatidylinositol-3-kinase (PI3K)-Akt axis, as miR-34a, suppresses PI3K, which regulates survivin mRNA expression *via* Akt activation (92). Last, miR-34a inhibits the Notch-1 signaling pathway, which in consequence downregulates its downstream target survivin (93).

The article "Dysregulation of Survivin-Targeting microRNAs in Autoimmune Diseases: New Perspectives for Novel Therapies" was retracted in 2023. Reason: concerns about the authorship.

Similarly, miR-203 is a survivin-targeting miRNA with an increased expression profile in RA synovial fibroblasts. It has been demonstrated that miR-203 may directly target survivin mRNA or the nuclear factor-kappa B (NF-κB) pathway, which can be hypothesized to down-regulate survivin expression (60–62) (**Figure 2**). Even so, other miRNAs with dysregulated expression patterns in RA patients, such as miR-335 and miR-485, have been identified to regulate survivin through direct interaction with its mRNA (7, 74, 94). However, further studies are required to determine the precise impact of these miRNAs on survivin expression in RA patients, leading to innovative targeted therapeutics for RA.

**Figure 2:** The survivin-miRNA axis is depicted schematically. Several survivin-targeting miRNAs regulate survivin expression either directly by binding to the 3′-UTR of survivin mRNA or indirectly by influencing the pathways that alter survivin expression as a downstream target. For example, miR-16 inhibits the p53/survivin signaling pathway, resulting in survivin downregulation, while miR-21 and miR-150 downregulate PTEN. PTEN inhibits Akt *via* the PI3k axis, NF-κB-dependent survivin upregulation occurs. Similarly, miR-203 and miR-16 regulate survivin expression by interacting with NF-κB. MiR-20 is another well-established survivin-targeting miRNA that inhibits SFMBT1 and regulates the TGF-β1/Survivin pathway. Moreover, miR-125 and miR-34a indirectly regulate survivin expression through interaction with STAT3 and E2F3, respectively. Conversely, miR-34a, miR-203, miR-16, miR-708, miR-485, and miR-335 specifically target the 3’ UTR of survivin mRNA and hence downregulate survivin expression. PTEN, Phosphatase and tensin homolog; Akt, Protein kinase B; NF-κB, Nuclear factor-kappa B; TGF-β, Transforming growth factor-beta; E2F3, Transcription Factor 3; STAT3, signal transducer and activator of transcription 3; 3′-UTRs, 3′-untranslated regions.

The article "Dysregulation of Survivin-Targeting microRNAs in Autoimmune Diseases: New Perspectives for Novel Therapies" was retracted in 2023. Reason: concerns about the authorship.

### Inflammatory *Bowel D*isease (IBD)

IBD, which comprises Crohn’s Disease (CD) and Ulcerative Colitis (UC), is a chronic inflammatory condition of the gastrointestinal tract with an intricate etiopathogenesis involving genetic predisposition, dysbiosis, increased intestinal permeability, and a dysregulated immune response. These factors lead to loss of tolerance to self-antigens and an overactive mucosal immune response against gut flora, which ultimately contributes to epithelial cell destruction (95). Immunopathological research has highlighted CD’s aberrant Th1 and Th17 responses, characterized by increased IL-12/IL-23 and IFN-γ/IL-17, respectively. In contrast, UC is characterized by the aberrant Th2 response and an excess release of IL-5/IL-13, which disproportionately impacts the colon (96). Collectively, the immunopathogenesis of the IBD primarily relies upon abnormally up-regulated proliferation and defective apoptosis regulation of CD4^+^ T cells. Although research into the molecular basis underlying this phenomenon is still in its infancy, the implication of survivin has been well investigated. A recent study has uncovered the high expression of survivin in CD4^+^ T cells from UC patients that binds to the FasL transcription factor, leading to dysregulated activation-induced cell death (AICD) in these cells (97). Survivin was also shown to be abundantly expressed in lamina propria T cells from CD patients compared to UC patients or healthy counterparts, which was suggested to engage with heat shock protein 90 (HSP90) and hinder the proteasomal degradation pathway of apoptotic machinery (51). Another case-control study found a substantial variation in survivin promoter polymorphism - 31C/G among IBD patients and their control counterparts, attributed to IBD susceptibility (98).

Several investigations have outlined miRNA dysregulation as an essential factor of IBD pathophysiology. As previously stated, miR-16 is a survivin-targeting miRNA that regulates survivin expression *via* interaction with p53. It has been shown to be up-regulated in the serum of IBD patients and to positively regulate the NF-κB pathway, which may be involved in regulating survivin expression (63, 64). Similarly, miR-21 has been reported to be excessively up-regulated in colon tissue and CD4^+^ T cells of patients with IBD (99). MiR-21 has been demonstrated to downregulate the phosphatase and tensin homolog deleted from chromosome Ten (PTEN), which is negatively associated with survivin expression (65, 66) (**Figure 2**).

The article "Dysregulation of Survivin-Targeting microRNAs in Autoimmune Diseases: New Perspectives for Novel Therapies" was retracted in 2023. Reason: concerns about the authorship.

In summary, survivin-targeting miRNAs play an essential part in IBD immunopathogenesis by enhancing survivin expression in CD4^+^ T cells, which compromises apoptosis regulation and leads to excessive autoreactive immune responses to gut flora, culminating in epithelium damage.

### Psoriasis

Psoriasis is a chronic inflammatory dermatosis characterized by the infiltration of inflammatory cells in the epidermis and dermis, leading to keratinocyte hyperproliferation and hyperkeratosis (100). In chronic psoriatic plaque lesions, DCs trigger T cell subsets (Th1, Th17, Th22) expansion and activation that release IFN-γ, IL-17, TNF-α, and IL-22 binding to their receptors on keratinocytes, rendering these cells hyperproliferative and resistant to apoptosis (101–103). The proliferative and antiapoptotic properties of keratinocytes in psoriasis have underpinned the plausibility of survivin involvement in the pathogenesis of psoriasis. In this way, several studies have evaluated survivin levels in patients with psoriasis. Survivin serum levels were considerably higher in psoriasis patients than controls (52).

Furthermore, psoriatic tissues have been demonstrated to express higher survivin mRNA than their control counterparts (104). In multiple studies, the molecular basis of survivin overexpression in psoriasis patients has been attributed to the NF-κB pathway. It was discovered that diffuse nuclear expression of NF-κB was significantly correlated with survivin up-regulation in psoriatic plaque (105). In accordance with these findings, dimethyl fumarate, an inhibitor of the NF-κB pathway, has been shown to enhance apoptosis by suppressing the NF-κB-induced upregulation of anti-apoptotic protein-encoding genes, including survivin (106). Aside from NF-κB, several pathways have been identified to regulate survivin expression in psoriasis patients. The Wnt/-Catenin and Wnt5a/Ca^2+^ pathways have been reported to enhance keratinocyte proliferation while suppressing apoptosis pathways in these cells by negatively regulating apoptosis-regulatory proteins such as survivin (107).

Several dysregulated miRNAs have been implicated in psoriasis pathogenesis by directly or indirectly targeting survivin expression. In this context, miR-20a-3p has been shown to have a low expression profile in psoriatic lesions and keratinocytes of psoriasis patients. *In vitro* studies revealed that overexpression of miR-20a-3p directly induces post-transcriptional suppression of SFMBT1, leading to transforming growth factor beta-1 (TGFβ1) and P-smad2/3 protein upregulation and survivin downregulation (67). Further, miR-125b has been demonstrated to be downregulated in keratinocytes of psoriasis patients, contributing to their enhanced proliferative status (108). Survivin is upregulated in keratinocytes *via* a positive feedback loop involving STAT3/SH3PXD2A-AS1/miR-125b/STAT3 (68) (**Figure 2**).

The article "Dysregulation of Survivin-Targeting microRNAs in Autoimmune Diseases: New Perspectives for Novel Therapies" was retracted in 2023. Reason: concerns about the authorship.

Collectively, enhanced proliferative state and impaired apoptosis regulation of keratinocytes in psoriasis might be attributed to dysregulation of survivin-targeting miRNAs, which could be a viable target for prospective targeted therapies.

### Systemic Lupus Erythematosus (SLE)

SLE is a complex multisystemic autoimmune condition marked by a loss of immunological tolerance to cellular, nuclear, and extracellular components. It developed autoantibodies directed against them, deposition of immune complexes, persistent inflammation, and tissue destruction (109). The pathogenesis of SLE is primarily associated with dysregulation of apoptotic debris disposal, which enhances nuclear antigen exposure and recognition by Toll-like receptors (TLRs), resulting in a significant infiltration of inflammatory cells. Infiltrated neutrophils play a central role in the immunopathogenesis of SLE, partly by releasing type 1 interferon (I-IFN) and partly by amplifying nuclear antigen exposure by forming extracellular neutrophil traps (NETosis), which leads to the recruitment of much more I-IFN-producing inflammatory cells, particularly plasmacytoid DCs. These cells enhance B cell autoreactivity and autoantibody production while also inducing aberrant T cell activation, further amplifying B cell autoreactivity and IL-17 production, causing tissue damage (110, 111). As aforementioned, survivin, an antiapoptotic molecule, is vital for immune cell homeostasis and plays a significant role in autoreactivity and apoptosis escape. Thus, aberrant survivin expression in immune cells involved in SLE pathogenesis might be critical in their hyperactivation and autoreactivity. However, survivin implication in SLE pathogenesis might be dissimilar to other autoimmune conditions. A recent study found that patients with SLE have lower serum survivin levels than their control counterparts (53). It is justified that clearance deficit is the primary driver of SLE pathogenesis, and low survivin level raises apoptosis in SLE, followed by triggered autoimmunity directed against autoantigens (112).

Until yet, the relevance of survivin-targeting miRNAs in SLE has received little attention, and more investigations are warranted. However, some evidence substantiates the implication of these miRNAs in SLE pathogenesis. As previously stated, miR-16 and miR-203 are survivin-regulating miRNAs that suppress survivin expression *via* various mechanisms. In contrast to RA, it has been demonstrated that serum levels of miR-16 and miR-203 are diminished in SLE patients compared to healthy controls (69, 70), indicating their likely participation in survivin downregulation in serum of patients with SLE. Furthermore, miR-20a is a survivin-targeting miRNA with decreased expression in SLE patients’ serum (69). According to research, miR-20a boosts NF-κB pathway activation by interacting with an NF-κB inhibitor, resulting in survivin upregulation (71). Also, like IBD, CD4^+^ T cells from SLE patients have an enhanced expression profile of miR-21, which interacts with PTEN to downregulate its expression and, as a consequence, induces survivin upregulation (66, 72).

The article "Dysregulation of Survivin-Targeting microRNAs in Autoimmune Diseases: New Perspectives for Novel Therapies" was retracted in 2023. Reason: concerns about the authorship.

Altogether, survivin-targeting miRNAs are postulated to contribute to SLE pathogenesis in two opposite directions. In apoptotic cells, these miRNAs downregulate anti-apoptotic survivin expression, which results in enhanced apoptosis; on the other hand, in autoreactive immune cells, survivin-targeting miRNAs contribute to survivin upregulation, enhancing their sustained activation and autoreactivity.

### Multiple *Sclerosis* (MS)

MS is a complex, chronic neurodegenerative condition characterized by autoreactive immune invasion, peripherally mediated inflammation, and persistent central nervous system (CNS)-compartmentalized inflammation, leading to demyelination and severe neurological complications (113). MS immunopathogenesis primarily relies on dysregulated Th1 and Th17 mediated autoreactive immunity triggered by environmental pathogens or other factors with antigenic sequences similar to those found in myelin, resulting in molecular mimicry and cross-reactivity with myelin. After that, the recruitment of immune cells leads to focal inflammation and CNS damage (114, 115). Although T cells are thought to be the primary contributors to MS immunopathogenesis, B cells play a significant role in the disease by priming T cells, enhancing brain-homing T cell autoproliferation, releasing pro-inflammatory cytokines, acting as a reservoir for Epstein-Barr virus (EBV), and producing autoantibodies against myelin antigens (116). As previously discussed, survivin is endowed with a regulative role in immune responses, implying that it may have a role in developing autoreactive immune responses in MS patients. Several studies have indicated that AICD in T cell subsets from MS patients is defective (117). In this context, analyses of T cells from MS patients outlined that these cells had an enhanced level of anti-apoptotic survivin, which contributes to the disease’s progression (54, 118, 119).

The article "Dysregulation of Survivin-Targeting microRNAs in Autoimmune Diseases: New Perspectives for Novel Therapies" was retracted in 2023. Reason: concerns about the authorship.

Recent research has established a link between dysregulation of survivin-targeting miRNAs and apoptotic resistance in CD4^+^ T cells derived from MS patients. Survivin mRNA and serum levels of survivin expression were inversely linked with miR-485 expression in CD4^+^ T cells (8). The same study also identified the downregulation of miR-708 in these cells compared to healthy controls (8). In this regard, several studies have discovered that miR-485 and miR-708 directly target the 3′-UTR of survivin mRNA and downregulate its production (74, 75); hence, miR-485 and miR-708 downregulation in CD4^+^ T cells contributes to survivin overexpression and thus defective apoptosis regulation. Similarly, miR-34a expression was lower in PBMCs from MS patients than healthy controls, and it is negatively associated with survivin mRNA expression and serum level (73). The mechanism by which this miRNA regulates survivin expression has already been discussed.

Overall, survivin’s significance in regulating the elimination of autoreactive immune cells has been well established, and several miRNAs have been discovered to regulate survivin expression in MS patients; however, understanding the precise mechanism of survivin-targeting miRNAs’ implication in MS pathogenesis and their promise as a target for the treatment of these patients warrants further investigations.

## Clinical Perspectives of Targeting Survivin-miRNA Axis as Master Regulator Route in Autoimmune Disease

Multiple survivin-targeting miRNAs have been established from the above concepts to implicate the etiopathogenesis of autoimmune diseases, suggesting the survivin-miRNA axis as a prospective target for therapeutic approaches. A plethora of anti-cancer therapeutic investigations have centered on miRNA-based strategies; however, their application in autoimmune conditions is still in its early stages, necessitating further research to develop and translate into a practical clinical approach. Nonetheless, the similar mechanistic participation of survivin-targeting miRNAs in establishing an over-proliferative and apoptosis-resistant state in malignant and autoreactive cells supports the plausibility of perspective approaches based on aberrant survivin-targeting miRNAs expression profiles in various autoimmune conditions. In this way, survivin-targeting miRNAs, whether overexpressed or down-expressed, can potentially be manipulated based on the targeted miRNA expression *via* miRNA replacement and antisense inhibition of mature miRNA (120).

miRNA replacement therapy has been extensively researched in anticancer therapies, holding the potential to restore the expression of miRNAs with a downregulated expression profile to achieve targeted expression (121). To that aim, cells with deficient miRNAs are directly transfected with synthetic miRNA mimics or vectors expressing the deficient miRNAs (122, 123). On the other hand, multiple strategies including, synthetic antisense oligonucleotides (ASOs), miRNA-masking oligonucleotides, miRNA sponges, and small-molecule inhibitors, have been employed to downregulate overexpressed miRNAs. ASOs bind to their target miRNAs in a specific and complementary manner, preventing them from interacting with their target mRNA. Similarly, miRNA-masking oligonucleotides disrupt miRNA-RNA interaction by interfering with the 3′-UTR of target mRNA. Additionally, miRNA sponges are short transcripts that mimic the 3′-UTR of target mRNA and bind to the miRNAs to suppress their function (124). On the other hand, small-molecule inhibitors can directly interact with the secondary motifs of pri- or pre-miRs or indirectly regulate the activity of miRNAs by interfering with their biogenesis (125).

The article "Dysregulation of Survivin-Targeting microRNAs in Autoimmune Diseases: New Perspectives for Novel Therapies" was retracted in 2023. Reason: concerns about the authorship.

Furthermore, it is demonstrated that modulating the microenvironment balance, whether through reduced or increased estrogen and 3,3’,5-triiodo-L-thyronine (T3), is a potential way of regulating miRNA expression. Given that estrogen and T3 may have a regulatory role in the expression of several survivin-targeting miRNAs such as miR-34 and miR-125, hormone therapy may benefit various autoimmune diseases (12, 126, 127).

Collectively, there is an imperative need to do preclinical and clinical research to validate the application of miRNA-based therapeutics to target the survivin-miRNA axis in autoimmune disease.

## Conclusion

Survivin, as a mitotic and anti-apoptotic factor, plays a vital role in the development and function of immune cells. In autoimmune diseases, aberrant survivin expression in over-proliferative and apoptosis-resistant cells has a remarkable role in disease development and progression. However, various miRNAs regulate survivin expression that exhibits dysregulated expression profiles in autoimmune conditions, which induce persistent and uncontrolled autoreactivity of immune cells and other cells involved in disease pathogenesis. These findings highlight the significant relevance of survivin-targeting miRNAs in autoimmune conditions and suggest the survivin-miRNA axis as a feasible therapeutic target that merits further research.

## Author Contributions

NS, AS, and AS: Conceptualization; Writing-original draft, Visualization. BB: Conceptualization. MS: Conceptualization; Resource. HM and MH: Writing-review & editing. FM: Visualization. SS: Project administration; Supervision. MJ: Project administration; Supervision, Resource. All authors contributed to the article and approved the submitted version.

The article "Dysregulation of Survivin-Targeting microRNAs in Autoimmune Diseases: New Perspectives for Novel Therapies" was retracted in 2023. Reason: concerns about the authorship.

## Funding

We have received a grant from the Immunology Research Center, Tabriz University of Medical Sciences, Tabriz, Iran (Grant No: 65139).

## Conflict of Interest

The authors declare that the research was conducted in the absence of any commercial or financial relationships that could be construed as a potential conflict of interest.

## Publisher’s Note

All claims expressed in this article are solely those of the authors and do not necessarily represent those of their affiliated organizations, or those of the publisher, the editors and the reviewers. Any product that may be evaluated in this article, or claim that may be made by its manufacturer, is not guaranteed or endorsed by the publisher.
